The article "The roles of ANRIL polymorphisms in coronary artery disease: a meta-analysis" was published in 2019. Journal: Biosci Rep.

# The roles of *ANRIL* polymorphisms in coronary artery disease: a meta-analysis

**DOI:** 10.1042/BSR20181559

**Published:** 2019-12-20

**Authors:** Lina Hu, Guoyi Su, Xia Wang

**Affiliations:** Guangdong Provincial Hospital of Chinese Medicine, The Second Clinical Medical College of Guangzhou University of Chinese Medicine, Guangzhou 510120, China

**Keywords:** Antisense non-coding RNA in the INK4 locus (ANRIL), Coronary artery disease (CAD), Gene polymorphisms, Meta-analysis

## Abstract

**Background:** The relationship between antisense non-coding RNA (ncRNA) in the INK4 locus (*ANRIL*) polymorphisms and coronary artery disease (CAD) remains inconclusive. Thus, we conducted this meta-analysis to better evaluate the roles of *ANRIL* polymorphisms in CAD. **Methods:** Systematic literature search of PubMed, Medline, and Embase was performed to identify potential relevant articles. Odds ratios (ORs) and 95% confidence intervals (CIs) were calculated to estimate the strength of association. **Results:** Fifteen studies were finally enrolled for analyses. Overall analyses suggested that rs1333040 (dominant model: *P*<0.0001; recessive model: *P*<0.0001; allele model: *P*<0.0001), rs1333049 (dominant model: *P*=0.02; allele model: *P*=0.02) and rs2383207 (additive model: *P*=0.004) polymorphisms were significantly associated with the risk of CAD. Further subgroup analyses showed that rs1333040, rs1333049, and rs2383207 polymorphisms were significantly correlated with the risk of CAD in East Asians, rs2383206 and rs10757274 polymorphisms were significantly correlated with the risk of CAD in West Asians, while rs2383206, rs10757274, and rs10757278 polymorphisms were significantly correlated with the risk of CAD in Caucasians. **Conclusion:** Our findings indicated that rs1333040, rs1333049, rs2383206, rs2383207, rs10757274, and rs10757278 polymorphisms might serve as genetic biomarkers of CAD in certain ethnicities.

## Introduction

Coronary artery disease (CAD), featured by narrowing or even occlusion of coronary arteries, is the primary cause of death and disability worldwide [1,2]. Until now, the exact pathogenic mechanism of CAD remains unclear. Nevertheless, mounting evidence supports that genetic factors are crucial for its occurrence and development. In the first place, family aggregation of CAD was not uncommon, and past twin studies showed that the heredity grade of CHD was over 50% [3,4]. In the second place, numerous genetic variants were found to be associated with an increased risk of CAD by previous genetic association studies, and screening of common causal variants was also shown to be a cost-efficient way to predict the individual risk of developing CAD [5,6]. In summary, these findings jointly indicated that genetic predisposition to CAD played a central part in its pathogenesis.

The article "The roles of ANRIL polymorphisms in coronary artery disease: a meta-analysis" was published in 2019. Journal: Biosci Rep.

Non-coding RNAs (ncRNAs) make up the vast majority of the human genome. Although ncRNAs do not encode proteins, it was evident that they play eminent roles in regulating expression levels of neighboring protein-encoding genes [7,8]. Therefore, dysregulation of ncRNAs may cause abnormal gene expression and give rise to the development of multiple diseases. Antisense ncRNA in the INK4 locus (*ANRIL*) is located on human chromosome 9p21, a region that has been repeated found to be associated with atherosclerosis and its related ischemia cardiovascular diseases like CAD [9]. Although the exact function of *ANRIL* is still unknown, it was shown that the expression levels of several neighboring protein-encoding genes like cyclin-dependent kinase inhibitors 2A (*CDKN2A*), *CDKN2B*, and methylthioadenosine phosphorylase (*MTAP*) were modulated by *ANRIL* [10]. Previous investigations demonstrated that the abovementioned proteins were abundantly expressed in atherosclerotic lesions, and they could promote atherosclerosis by impacting vascular remodeling, thrombogenesis, and plaque stability [9,10]. Hence, it is biologically plausible that these *ANRIL* polymorphisms may also be involved in atherosclerotic-related diseases like CAD. So far, some pilot studies already investigated potential correlations between *ANRIL* gene polymorphisms and the risk of CAD. But the results of these studies were controversial. Thus, we performed the present meta-analysis to better evaluate the roles of *ANRIL* polymorphisms in CAD.

## Materials and methods

### Literature search and inclusion criteria

This meta-analysis complied with the Preferred Reporting Items for Systematic Reviews and Meta-analyses (PRISMA) guidelines [11]. Potentially related literatures that were published before September 2018 were retrieved from PubMed, Medline, and Embase using the following combination of keywords: (*antisense noncoding RNA in the INK4 locus* OR *CDKN2B antisense RNA* OR *ANRIL* OR *CDKN2B-AS long non-coding RNA*) AND (polymorphism OR variant OR mutation OR genotype OR allele) AND (coronary heart disease OR coronary artery disease OR angina pectoris OR acute coronary syndrome OR myocardial infarction).

The references of retrieved articles were also screened to identify other potentially relevant studies.

To test the research hypothesis of this meta-analysis, included studies must meet all the following criteria: (i) case–control study on correlations between *ANRIL* polymorphisms and the risk of CAD; (ii) provide genotypic frequencies of investigated *ANRIL* polymorphisms in cases and controls; and (iii) full text in English available.

The article "The roles of ANRIL polymorphisms in coronary artery disease: a meta-analysis" was published in 2019. Journal: Biosci Rep.

Studies were excluded if one of the following criteria was fulfilled: (i) not relevant to *ANRIL* polymorphisms and CAD; (ii) case reports or case series; and (iii) abstracts, reviews, comments, letters, and conference presentations.

For duplicate publications, we only included the study with the largest sample size for analyses.

### Data extraction and quality assessment

The following data were extracted from included studies: (i) name of the first author; (ii) publication time; (iii) country and ethnicity; (iv) sample size; and (v) genotypic distributions of *ANRIL* polymorphisms in cases and controls. Additionally, the probability value (*P*-value) of Hardy–Weinberg equilibrium (HWE) was also calculated. When necessary, we wrote to the corresponding authors for raw data. We used the Newcastle–Ottawa scale (NOS) to assess the quality of eligible studies [12]. This scale has a score range of 0–9, and studies with a score of more than 7 were thought to be of high quality. Two reviewers conducted data extraction and quality assessment independently. Any disagreement between two reviewers was solved by discussion until a consensus was reached.

### Statistical analyses

All statistical analyses were conducted with Review Manager Version 5.3.3 (The Cochrane Collaboration, Software Update, Oxford, United Kingdom). Odds ratios (ORs) and 95% confidence intervals (CIs) were calculated to estimate strength of associations between *ANRIL* polymorphisms and the risk of CAD in all possible genetic models, and *P*-values ≤0.05 were considered to be statistically significant. Between-study heterogeneities were evaluated with *I^2^* statistic. If *I^2^* was greater than 50%, random-effect models (REMs) would be used to pool the data. Otherwise, fixed-effect models (FEMs) would be employed for synthetic analyses. Subgroup analyses by ethnicity of participants were subsequently performed. Sensitivity analyses were conducted to examine the stability of synthetic results. Funnel plots were used to assess publication bias.

## Results

### Characteristics of included studies

We found 105 potential relevant articles. Amongst these articles, a total of 15 eligible studies were finally included for synthetic analyses (see Figure 1). The NOS score of eligible articles ranged from 7 to 8, which indicated that all included studies were of high quality. Baseline characteristics of included studies are shown in Table 1.

**Figure 1:** Flowchart of study selection for the present study

**Table 1:** The characteristics of included studies for *ANRIL* polymorphisms and CAD

First author, year	Country	Ethnicity	Type of disease	Sample size	Genotype distribution		*P*-value for HWE	NOS score
					Cases	Controls		
**rs1333040**					TT/TC/CC			
Kumar (2011)	India	West Asian	CAD	300/423	147/116/37	175/182/66	0.107	7
Lin (2011)	Taiwan	East Asian	MI	411/1352	228/156/27	649/573/130	0.829	7
Qi (2012)	China	East Asian	MI	142/192	91/44/7	90/93/9	0.013	8
Scheffold (2011)	Germany	Caucasian	MI	976/3532	292/503/181	889/1750/893	0.590	7
Zhao (2016)	China	East Asian	CAD	456/683	236/184/36	336/293/54	0.370	7
**rs1333049**					GG/GC/CC			
Ahmed (2013)	Pakistan	West Asian	MI	294/290	65/166/63	87/180/23	<0.001	8
Çakmak (2015)	Turkey	Caucasian	CAD	220/240	54/120/46	85/115/40	0.917	7
Haslacher (2016)	Austria	Caucasian	MI	493/431	139/236/118	112/222/97	0.514	7
Lin (2011)	Taiwan	East Asian	MI	423/1361	100/218/105	395/655/311	0.213	7
Qi (2012)	China	East Asian	MI	142/192	42/79/21	50/99/43	0.651	8
Scheffold (2011)	Germany	Caucasian	MI	976/999	212/518/246	292/502/205	0.688	7
Yang (2018)	China	East Asian	CAD	542/549	162/269/111	176/273/100	0.743	8
**rs2383206**					AA/AG/GG			
Abdullah (2008)	U.S.A.	Caucasian	CAD	310/560	56/124/130	143/279/138	0.934	8
Kumar (2011)	India	West Asian	CAD	309/434	112/143/54	116/224/94	0.467	7
Scheffold (2011)	Germany	Caucasian	MI	976/9053	183/521/272	2489/4583/1981	0.017	7
Shendy (2017)	Egypt	West Asian	CAD	100/50	51/42/7	23/15/12	0.009	8
Zhou (2008)	China	East Asian	CAD	1360/1360	373/600/387	382/669/309	0.623	8
**rs2383207**					GG/GA/AA			
Abdullah (2008)	U.S.A.	Caucasian	CAD	310/560	139/121/50	147/277/136	0.807	8
Çakmak (2015)	Turkey	Caucasian	CAD	220/240	83/101/36	102/118/20	0.079	7
Chen (2009)	China	East Asian	CAD	212/232	107/69/36	71/114/47	0.920	8
El-Menyar (2015)	Egypt	West Asian	CAD	236/152	146/77/12	84/58/10	0.998	7
Kumar (2011)	India	West Asian	CAD	301/424	137/124/40	174/190/60	0.485	7
Lin (2011)	Taiwan	East Asian	MI	415/1349	214/162/39	568/609/172	0.660	7
Qi (2012)	China	East Asian	MI	142/192	78/55/9	82/93/17	0.192	8
Scheffold (2011)	Germany	Caucasian	MI	976/3532	183/519/274	1016/1770/746	0.628	7
Yang (2018)	China	East Asian	CAD	540/548	247/236/57	244/251/53	0.317	8
Zhou (2008)	China	East Asian	CAD	1360/1360	702/520/138	592/605/163	0.659	8
**rs10757274**					GG/GA/AA			
Abdullah (2008)	U.S.A.	Caucasian	CAD	310/560	61/119/130	156/283/121	0.728	8
El-Menyar (2015)	Egypt	West Asian	CAD	309/434	122/133/54	143/206/85	0.486	7
Kumar (2011)	India	West Asian	CAD	310/439	116/135/59	144/210/85	0.591	7
Mafi Golchin (2017)	Iran	West Asian	CAD	103/102	40/47/16	22/51/29	0.962	8
Scheffold (2011)	Germany	Caucasian	MI	976/9053	208/515/253	2752/4543/1758	0.131	7
Zhao (2016)	China	East Asian	CAD	291/385	82/137/72	130/188/67	0.945	7
**rs10757278**					GG/GA/AA			
Abdullah (2008)	U.S.A.	Caucasian	CAD	310/560	59/135/116	159/294/107	0.162	8
Chen (2009)	China	East Asian	CAD	212/232	107/69/36	71/114/47	0.920	8
El-Menyar (2015)	Egypt	West Asian	CAD	309/427	89/142/78	103/214/110	0.957	7
Scheffold (2011)	Germany	Caucasian	MI	976/718	211/522/243	224/366/128	0.308	7
Shendy (2017)	Egypt	West Asian	CAD	100/50	37/45/18	13/18/19	0.057	8

*P*-values ≤0.05 were considered to be statistically significant. Abbreviation: MI, myocardial infarction.

The article "The roles of ANRIL polymorphisms in coronary artery disease: a meta-analysis" was published in 2019. Journal: Biosci Rep.

### Overall and subgroup analyses

To investigate potential correlations between *ANRIL* polymorphisms and the risk of CAD, five studies about rs1333040 polymorphism, seven studies about rs1333049 polymorphism, five studies about rs2383206 polymorphism, ten studies about rs2383207 polymorphism, six studies about rs10757274 polymorphism, and five studies about rs10757278 polymorphism were enrolled for analyses.

Significant associations with the risk of CAD were detected for rs1333040 (dominant model: *P*<0.0001, OR = 1.30, 95% CI: 1.17–1.44; recessive model: *P*<0.0001, OR = 0.71, 95% CI: 0.62–0.82; allele model: *P*<0.0001, OR = 1.25, 95% CI: 1.16–1.34), rs1333049 (dominant model: *P*=0.02, OR = 0.81, 95% CI: 0.67–0.96; allele model: *P*=0.02, OR = 0.86, 95% CI: 0.76–0.98), and rs2383207 (additive model: *P*=0.004, OR = 0.80, 95% CI: 0.69–0.93) polymorphisms in overall analyses.

Further subgroup analyses according to ethnicity of participants revealed that rs1333040 (dominant model and allele model), rs1333049 (recessive model), and rs2383207 (all genetic models) polymorphisms were significantly correlated with the risk of CAD in East Asians, rs2383206 (dominant model and allele model) and rs10757274 (dominant model and allele model) polymorphisms were significantly correlated with the risk of CAD in West Asians, while rs2383206 (dominant model, recessive model, and allele model), rs10757274 (dominant model, recessive model, and allele model) and rs10757278 (dominant model, recessive model, and allele model) polymorphisms were significantly correlated with the risk of CAD in Caucasians (see Table 2).

**Table 2:** Overall and subgroup analyses for *ANRIL* polymorphisms and CAD

Polymorphisms	Population	Sample size	Dominant comparison		Recessive comparison		Additive comparison		Allele comparison	
			*P*-value	OR (95% CI)	*P*-value	OR (95% CI)	*P*-value	OR (95% CI)	*P*-value	OR (95% CI)
**rs1333040**	Overall	2285/6182	**<0.0001**	**1.30 (1.17–1.44)**	**<0.0001**	**0.71 (0.62–0.82)**	0.12	0.85 (0.69**–**1.04)	**<0.0001**	**1.25 (1.16–1.34)**
	East Asian	1009/2227	**0.03**	**1.37 (1.04–1.80)**	0.18	0.82 (0.61**–**1.09)	0.06	0.76 (0.57**–**1.01)	**0.001**	**1.22 (1.08–1.38)**
**rs1333049**	Overall	3090/4062	**0.02**	**0.81 (0.67–0.96)**	0.08	1.24 (0.98**–**1.57)	0.35	1.05 (0.95**–**1.15)	**0.02**	**0.86 (0.76–0.98)**
	Caucasian	1689/1670	0.37	0.85 (0.60**–**1.20)	0.93	1.02 (0.69**–**1.51)	0.32	1.10 (0.91**–**1.31)	0.59	0.93 (0.72**–**1.20)
	East Asian	1107/2102	0.16	0.82 (0.61**–**1.09)	**0.02**	**1.19 (1.03–1.38)**	0.31	1.07 (0.94**–**1.20)	0.06	0.87 (0.75**–**1.01)
**rs2383206**	Overall	3055/11457	0.60	0.91 (0.64**–**1.29)	0.33	1.18 (0.84**–**1.65)	0.36	0.90 (0.72**–**1.13)	0.45	0.91 (0.72**–**1.16)
	Caucasian	1286/9613	**<0.0001**	**0.61 (0.53–0.71)**	**0.02**	**1.71 (1.08–2.71)**	0.61	0.88 (0.53**–**1.45)	**0.0002**	**0.68 (0.56–0.84)**
	West Asian	409/484	**0.006**	**1.49 (1.12–1.99)**	0.19	0.47 (0.15**–**1.46)	0.83	1.08 (0.53**–**2.19)	**0.002**	**1.36 (1.12–1.65)**
**rs2383207**	Overall	4712/8589	0.09	1.29 (0.96**–**1.72)	0.66	0.94 (0.73**–**1.22)	**0.004**	**0.80 (0.69–0.93)**	0.15	1.17 (0.95**–**1.45)
	Caucasian	1506/4332	0.97	1.02 (0.42**–**2.47)	0.58	1.21 (0.62**–**2.35)	0.48	0.88 (0.61**–**1.26)	0.94	0.98 (0.55**–**1.75)
	East Asian	2669/3681	**0.0003**	**1.45 (1.18–1.79)**	**0.03**	**0.83 (0.71–0.98)**	**<0.0001**	**0.77 (0.69–0.85)**	**0.0005**	**1.28 (1.11–1.48)**
	West Asian	537/576	0.08	1.24 (0.97**–**1.58)	0.57	0.89 (0.61**–**1.32)	0.15	0.84 (0.65**–**1.07)	0.12	1.16 (0.96**–**1.39)
**rs10757274**	Overall	2299/10973	0.89	0.98 (0.69**–**1.39)	0.27	1.23 (0.85**–**1.76)	0.15	0.86 (0.70**–**1.06)	0.89	0.98 (0.69**–**1.39)
	Caucasian	1286/9613	**<0.0001**	**0.62 (0.54–0.72)**	**0.03**	**1.92 (1.08–3.42)**	0.54	0.83 (0.46**–**1.50)	**0.001**	**0.65 (0.50–0.84)**
	West Asian	722/975	**0.003**	**1.36 (1.11–1.67)**	0.17	0.84 (0.66**–**1.08)	0.08	0.84 (0.69**–**1.02)	**0.04**	**1.28 (1.01–1.62)**
**rs10757278**	Overall	1907/1987	0.81	1.09 (0.63**–**1.87)	0.72	1.10 (0.67**–**1.81)	0.24	0.83 (0.61**–**1.13)	0.87	1.03 (0.70**–**1.52)
	Caucasian	1286/1278	**<0.0001**	**0.60 (0.50–0.73)**	**0.008**	**1.95 (1.19–3.19)**	0.61	0.89 (0.57**–**1.39)	**<0.0001**	**0.65 (0.52–0.81)**
	West Asian	409/477	0.06	1.33 (0.98**–**1.80)	0.35	0.63 (0.24**–**1.66)	0.54	0.92 (0.70**–**1.20)	0.22	1.37 (0.83**–**2.27)

The values in bold represent that there are statistically significant differences between cases and controls. *P*-values ≤0.05 were considered to be statistically significant. Abbreviation: MI, myocardial infarction.

The article "The roles of ANRIL polymorphisms in coronary artery disease: a meta-analysis" was published in 2019. Journal: Biosci Rep.

### Sensitivity analyses

We performed sensitivity analyses by excluding studies that deviated from HWE. No alterations of results were detected in sensitivity analyses, which suggested that our findings were statistically reliable.

### Publication biases

Publication biases were evaluated with funnel plots. We did not find obvious asymmetry of funnel plots in any comparisons, which indicated that our findings were unlikely to be impacted by severe publication biases.

## Discussion

To the best of our knowledge, this is so far the most comprehensive meta-analysis on correlations between *ANRIL* polymorphisms and the risk of CAD. The overall analyses suggested that rs1333040, rs1333049, and rs2383207 polymorphisms were significantly associated with CAD risk in overall population. Further subgroup analyses revealed that rs1333040, rs1333049, and rs2383207 polymorphisms were significantly correlated with the risk of CAD in East Asians, rs2383206 and rs10757274 polymorphisms were significantly correlated with the risk of CAD in West Asians, while rs2383206, rs10757274, and rs10757278 polymorphisms were significantly correlated with the risk of CAD in Caucasians.

There are several points that need to be addressed about this meta-analysis. First, the exact function of *ANRIL* is still unclear, and therefore the underlying mechanisms of our positive findings need to be elucidated by future investigations. Second, the pathogenic mechanism of CAD is highly complex, and therefore it is unlikely that a single gene polymorphism can significantly contribute to its development. As a result, to better illustrate potential correlations of certain gene polymorphisms with CAD, we strongly recommend further studies to perform haplotype analyses and explore potential gene–gene interactions. Thirdly, according to a previous investigation, subjects carrying mutant allele of rs1333049 polymorphism had elevated TC, TG and LDL-C levels, and this may partially explain the observed significant correlation between this polymorphism and the risk of CAD. For other investigated polymorphisms, however, future studies are needed to investigate whether these polymorphisms are correlated with clinical and biochemical parameters of CAD [13].

As with all meta-analysis, the present study certainly has some limitations. First, our results were derived from unadjusted analyses, and lack of further adjusted analyses for age, gender, and co-morbidity conditions may impact the reliability of our findings [14]. Second, obvious heterogeneities were found in several subgroups, which indicated that the controversial results of included studies could not be fully explained by differences in ethnic background and type of disease, and other baseline characteristics of participants may also contribute to between-study heterogeneities [15]. Third, associations between *ANRIL* polymorphisms and CAD may also be modified by gene-gene and gene-environmental interactions. However, most eligible studies did not consider these potential interactions, which impeded us to perform relevant analyses accordingly [16]. On account of abovementioned limitations, our findings should be cautiously interpreted.

The article "The roles of ANRIL polymorphisms in coronary artery disease: a meta-analysis" was published in 2019. Journal: Biosci Rep.

## Conclusion

In conclusion, our meta-analysis suggested that rs1333040, rs1333049, rs2383206, rs2383207, rs10757274, and rs10757278 polymorphisms might serve as genetic biomarkers of CAD in certain ethnicities. However, further well-designed studies are still warranted to confirm our findings.

## Abbreviations

ANRIL: antisense non-coding RNA in the INK4 locus
CAD: coronary artery disease
CI: confidence interval
HWE: Hardy–Weinberg equilibrium
ncRNA: non-coding RNA
NOS: Newcastle–Ottawa scale
OR: odds ratio
